The article "Fetal and Neonatal Middle Cerebral Artery Hemodynamic Changes and Significance under Ultrasound Detection in Hypertensive Disorder Complicating Pregnancy Patients with Different Severities" was published in 2022. Journal: Comput Math Methods Med.

# Fetal and Neonatal Middle Cerebral Artery Hemodynamic Changes and Significance under Ultrasound Detection in Hypertensive Disorder Complicating Pregnancy Patients with Different Severities

**DOI:** 10.1155/2022/6110228

**Published:** 2022-06-28

**Authors:** Pei Zhou, Yi Sun, Yongpan Tan, Yanru An, Xingxing Wang, Lufang Wang

**Affiliations:** Department of Ultrasound, The Fourth Hospital of Shijiazhuang, Shijiazhuang, 050000 Hebei, China

## Abstract

Colour Doppler ultrasound was applied for monitoring the hemodynamic parameters of fetal uterine artery (UtA), umbilical artery (UA), and middle cerebral artery (MCA) during pregnancy. In hypertension disease complicating pregnancy, these hemodynamic measures and their therapeutic applicability value were reviewed (HDCP). 120 singleton pregnant women were chosen, with 40 cases of mild preeclampsia (mild group), 40 cases of severe preeclampsia (severe group), and 40 normal control pregnant women (control group). The hemodynamic parameters of UtA, MCA, and UA were monitored in the three groups, including pulsatility index (PI), resistance index (RI), and the systolic/diastolic velocity (S/D). The parameters PI, RI, S/D, and venous catheter shunt rate (Qdv/Quv) of UtA and UA in the severe group were higher than those in the normal group and the mild group, showing the differences statistically significant (*P* < 0.05). The PI, RI, and S/D of MCA in the severe group were lower than those in the normal group and the mild group (*P* < 0.05). The changing trends of PI, RI, and S/D in the severe group were all first increased and then decreased in the early, middle, and later pregnancy (*P* < 0.05). The area under the curve (AUC) was 0.98 in the receiver operating characteristic (ROC) curve created using a combination of hemodynamic measures and pregnancy outcomes, and the sensitivity and specificity for predicting bad outcomes were 94.7 percent and 96.4 percent, respectively. Colour Doppler ultrasound may accurately detect changes in the PI, RI, and S/D of UtA, MCA, and UA in pregnant women and serve as a reference for determining the intrauterine state of the fetuses and predicting bad pregnancy outcomes. In particular, the parameters in later pregnancy were higher worthy of diagnostic value for adverse pregnancy outcomes. The combination of various parameters could make an improvement of the diagnostic accuracy and provide a basis for guiding treatment as well as determining the optimal timing of delivery.

## 1. Introduction

Hypertensive disorder complicating pregnancy (HDCP) is a group of diseases that coexist with pregnancy and elevated blood pressure, with an incidence of about 5% to 12%. It seriously affects the health of mothers and fetuses and is one of the important causes of maternal and fetal death [1–3]. The common methods for monitoring fetal intrauterine status include fetal movement counting, electronic fetal heart rate monitoring, fetal scalp blood gas analysis, fetal electrocardiogram, ultrasound, and amnioscopy. With ultrasound, not only the intrauterine growth of the fete but also the fetal position, placental position, amniotic fluid volume, and placental maturity can be determined; it is the most common imaging method in obstetrics [4, 5]. As colour Doppler flow imaging (CDFI) is combined with conventional two-dimensional ultrasound, the distribution of blood flow can be displayed, and the velocity of blood flow can be quantitatively measured. Thus, the distribution and passages of blood flow in blood vessels are shown more comprehensively [6].

The article "Fetal and Neonatal Middle Cerebral Artery Hemodynamic Changes and Significance under Ultrasound Detection in Hypertensive Disorder Complicating Pregnancy Patients with Different Severities" was published in 2022. Journal: Comput Math Methods Med.

Blood flow of umbilical artery (UA) has a wide range of applications clinically. By monitoring fetal UA blood flow parameters, placental blood perfusion and placental peripheral microcirculation resistance are evaluated, which is to judge fetal intrauterine status and predict pregnancy outcome [7–9]. The uterine artery (UtA) is the main blood vessel for blood circulation between the uterus and the placenta and is a crucial bridge between the fete and the mother. Both the diameter of the UtA and the blood flow velocity increase to meet the blood supply for the growth and development of the fetuses [10]. The fetal MCA expands to the internal carotid artery, and its oxygen supply occupies about 80% of the entire brain. Since the fetal brain is the most sensitive to intrauterine hypoxia, monitoring the blood flow parameters of the MCA can reflect the developmental status of fetal cerebral circulation directly, having a certain clinical value in assessing fetal intrauterine conditions and predicting pregnancy outcomes [11–13]. By detecting the blood flow parameters pulsatility index (PI), resistance index (RI), and the ratio of systolic peak velocity to diastolic end velocity (S/D) of fetal-related blood vessels like UtA, MCA, and UA, an objective basis can be obtained for determining the intrauterine status of the fetuses, guiding clinical treatment, and predicting pregnancy outcomes [14–17].

The blood flow parameters UtA, MCA, and UA in 120 pregnant women with singleton pregnancy were monitored and analysed in this research. It was aimed at the changes in blood flow parameters of UtA, MCA, and UA in HDCP patients and their correlation with pregnancy outcomes. It was expected to give a diagnostic basis for clinical application. The later-stage markers demonstrated a higher diagnostic value for negative pregnancy outcomes. All of the parameters together could increase diagnostic accuracy and offer a foundation for guiding treatment and identifying the ideal delivery time. The disadvantages of this study were that the measurements of several parameters might be affected by frequent fetal movement. The angle of sampling between the sound beam and the blood flow should be exact, and there may be minor mistakes.

The article "Fetal and Neonatal Middle Cerebral Artery Hemodynamic Changes and Significance under Ultrasound Detection in Hypertensive Disorder Complicating Pregnancy Patients with Different Severities" was published in 2022. Journal: Comput Math Methods Med.

The arrangements of the paper are as follows: Section 2 discusses the materials and methods.  Section 3 describes the results and discussion.  Section 4 examines the sensitivity and specificity of the combination of all parameters in diagnosing adverse pregnancy outcomes.  Section 5 concludes the article.

## 2. Materials and Methods

### 2.1. Research Objects

120 pregnant women were chosen as they went to the Fourth Hospital of Shijiazhuang for prenatal examination from November 2019 to December 2021. They had the singleton pregnancy at 32-34 weeks, including 40 cases with mild preeclampsia (mild group), 40 with severe eclampsia (severe group), and 40 normal pregnant women (control group). All cases were followed up to the end of their pregnancy. Their age ranged from 22 to 35 years old, with a mean value of 28.45 ± 2.36 years old. The gestational age was varied from 28 to 40 weeks, with 35.42 ± 4.3 weeks on average. Mild and severe preeclampsia in these cases conformed to the classification of HDCP in the 8th edition of Obstetrics and Gynecology [18]. This research had been approved by the Medical Ethics Committee of the Fourth Hospital of Shijiazhuang, and the patients and their families were informed about the research situation and signed the informed consents.

Inclusion criteria were listed as below.

1. Pregnant women went with the complete medical records, went for obstetric examination regularly, and received institutional delivery
2. They were health previously, with no smoking, alcohol abuse, and other bad habits
3. Their menstruation was regular, and the last menstrual period was clear; under early pregnancy ultrasound examination, the fetal size and menopause cycle were matched
4. They had no special medication history during pregnancy, and the fetuses got no congenital developmental malformation

The following were the exclusion criteria.

1. Ultrasound examination revealed fetal congenital abnormality or abnormal placenta
2. Ultrasound examination showed there were twins or multiples
3. The patients were accompanied with genital malformations or genital diseases
4. The patients had an acute infectious disease
5. They had a history of lower abdominal and pelvic surgery in the past
6. Patients went with obesity

### 2.2. Examination Methods

The probe frequency was 3.5 MHz, the sample volume was 2 mm, and the angle between the sound beam and blood flow was 30° using the Philips-IU22 full digital colour Doppler ultrasound diagnostic apparatus made in the Netherlands. Before the examination, all pregnant women emptied their urine and underwent routine obstetric ultrasound examination in the supine position. The fetal biparietal diameter (BPD), head circumference (HC), abdominal circumference (AC), femoral length (FL), and more growth indexes were examined. The fetal position and placental position were observed, and fetal heart rate, amniotic fluid volume, and more were monitored. After routine obstetric ultrasound examination, CDFI was performed for the measurement of the blood flow parameters PI, RI, and S/D of UtA, MCA, and UA and the maximum flow rate (V1) and inner diameter (D1) of umbilical vein (UV), as well as the maximum flow rate (V2) and inner diameter (D2) of ductus venosus (DV). All these were measured independently by the same experienced sonographer.

The article "Fetal and Neonatal Middle Cerebral Artery Hemodynamic Changes and Significance under Ultrasound Detection in Hypertensive Disorder Complicating Pregnancy Patients with Different Severities" was published in 2022. Journal: Comput Math Methods Med.

The blood flow volume of UV (Quv), the ductus-venous blood flow volume (Qdv), and the venous catheter shunt rate (Qdv/Quv) were calculated, respectively, as follows.

(1) $$\begin{array}{c} \text{Quv}=0.5\times \text{V}1\times \pi \times {\left(\frac{\text{D}1}{2}\right)}^{2}, \end{array}$$

(2) $$\begin{array}{c} \text{Qdv}=0.5\times \text{V}2\times \pi \times {\left(\frac{\text{D}2}{2}\right)}^{2}, \end{array}$$

(3) $$\begin{array}{c} \text{Venous catheter shunt rate}=\frac{\text{Qdv}}{\text{Quv}}. \end{array}$$

### 2.3. Detection of Blood Flow Parameters of UtA, MCA, and UA

First, two-dimensional ultrasound was applied to display UtA on both sides of the junction of the uterus and cervix through the abdomen. Then, CDFI was performed for the blood flow signal of UtA. 1-2 cm away from the internal iliac artery, the site in UtA was taken as the sampling point. The sample volume was set at 2 mm, and the angle between the sound beam and the blood flow was set at 30 degrees. Five or more distinct and stable characteristic spectra were collected before the image was locked.

The standard section for BPD measurement was chosen, and the probe moved along the BPD section toward the skull base. The large sphenoid bone was found between the anterior and middle cranial fossa, and CDFI was used for displaying the blood flow in the circle of Willis. Additionally, MCA originating from the left and right sides of the circle of Willis was also displayed. The midsection of the MCA was taken as the sampling point, the sampling volume was set to 2 mm, and the angle between the blood flow direction the sound beam was <60°. The images were frozen after the obtainment of 5 or more clear and stable characteristic spectra.

The article "Fetal and Neonatal Middle Cerebral Artery Hemodynamic Changes and Significance under Ultrasound Detection in Hypertensive Disorder Complicating Pregnancy Patients with Different Severities" was published in 2022. Journal: Comput Math Methods Med.

The free umbilical cord close to the placenta and not tortuous and knotted was selected, and the inside of the UA was the sampling point. With the sampling volume of 2 mm and the angle between the sound beam direction and the blood flow direction <30°, the images turned to be frozen after at least 5 clear and stable characteristic spectra were worked out.

The instrument measured RI, PI, and S/D of UtA, MCA, as well as UA automatically, each parameter was measured 3 times, and the mean value was taken and recorded.

### 2.4. Evaluation Criteria for Adverse Pregnancy Outcomes

Premature birth was defined as a delivery with the gestation over 28 weeks but less than 37 weeks. The Apgar score was a scoring system of 5 signs after birth, including heart rate, breathing, muscular tension, laryngeal reflex, and skin colour. Fetal growth restriction (FGR) was the impaired fetal growth potential, and the fetal weight estimated was less than the 10% of that with the same gestational age.

Diagnostic criteria for fetal intrauterine distress (FIUD) were explained as follows.

1. Fetal movement decreased or disappeared: the fetal movement counting < 10 times/2 h or got a decrease of 50%, which indicated the possibility of fetal hypoxia
2. Abnormal nonstress test results also indicated the possibility of fetal hypoxia, but the false positive rate was high; thus, it is needed to be reviewed
3. For the fetal biophysical score, 5-6 points indicated a suspected fetal hypoxia
4. Abnormal blood flow was presented in fetal CDFI: the ratio value of S/D increased, indicating insufficient placental blood perfusion and fetal hypoxia

### 2.5. Pregnancy Outcomes in Follow-Ups

When premature birth, FIUD, FGR, or neonatal asphyxia occurred, a poor pregnancy outcome was identified. In the follow-ups of perinatal prognosis, it was known whether there was a FIUD, neonatal asphyxia, FGR, and delivery gestational age. The perinatal outcomes of pregnant women were followed up; related indexes, maternal weeks at delivery, neonatal weight, pH value of UA, 5 min Apgar score, and placental weight, were recorded.

Adverse perinatal outcomes were divided into mild ones and the severe ones. Mild adverse outcomes included premature birth, pH of UA < 7.20, and birth weight < 2.5 kg. Severe adverse outcomes included intrauterine stillbirth, fetal death after birth, birth weight < 1.5 kg, and Apgar score ≤ 7.5 minutes after the birth.

### 2.6. Statistical Processing

All the data in this work were expressed as mean ± standard deviation ($\bar{x}\pm s$), and SPSS 19.0 was used for data analysis. Pairwise comparisons were performed using *t* test, and comparisons between or among groups were made using one-way analysis of variance. Logistic binary regression was used for the analysis of the related factors of poor perinatal prognosis. If *P* < 0.05, the difference was thought to be statistically significant.

The article "Fetal and Neonatal Middle Cerebral Artery Hemodynamic Changes and Significance under Ultrasound Detection in Hypertensive Disorder Complicating Pregnancy Patients with Different Severities" was published in 2022. Journal: Comput Math Methods Med.

## 3. Results and Discussion

### 3.1. Comparison of Mean Age and Gestational Age among Three Groups

There was not a significant difference in the mean age and mean gestational age among the three groups (*P* > 0.05), as listed in Table 1.

### 3.2. Blood Flow Spectra of Fetal UtA, MCA, and UA

The Doppler ultrasound spectral waveform of UtA was characterized by high resistance and low diastolic components in early pregnant women, and it was hump-shaped in the diastolic phase (two-peak continuous spectrum). In HDCP patients, intrauterine hypoxia was observed; diastolic notch was in UtA, which is presented in Figure 1.

For the measurement of fetal MCA, the Doppler sampling volume was in the middle of the artery. In the standard BPD section, the probe was moved parallel to the fetal skull base until the paired greater wings of sphenoid bone appeared between the anterior and the middle cranial fossae. CDFI showed the arterial ring of Willis; MCA originated from the left and right sides of the middle of the arterial ring and runs to the brain bilaterally, deviating to the frontal direction slightly. As shown in Figure 2, the blood flow resistance of fetal MCA in HDCP patients was lowered. The placental resistance was reflected in the blood flow of UA, and the partial diastolic blood flow spectrum of the fetal UA was absent or inverted in HDCP patients, as shown in Figure 3.

With the widespread use of colour Doppler ultrasound in prenatal diagnosis in recent years, clinical research in obstetrics and gynecology has gradually focused on the relationship between maternal and fetal ultrasound blood flow parameters, as well as the occurrence and progression of adverse pregnancy outcomes. Ultrasound detection indices can now be used as supplemental indices for HDCP diagnosis and treatment [19–21]. Abnormal UA spectrum is associated with placental 3rd-grade villous stem occlusion. With the development of the disease, the structure of the placental villi vessels changes, and the number of placental 3rd-grade villous stem arterioles decreases notably. The interstitial fibrosis worsens, and fibrous material is deposited, reducing the volume of fetal placental blood circulation and impeding fetal growth and development. Rubin et al. [22] pointed out that venous blood flow was reduced in fetuses with abnormal Doppler spectra of UA significantly. In the waveform of DV, the degree of downward deflection is proportional to the risk of fetal death or multisystem organ failure. Studies have shown that abnormal DV waveforms are strongly associated with fetal death.

The article "Fetal and Neonatal Middle Cerebral Artery Hemodynamic Changes and Significance under Ultrasound Detection in Hypertensive Disorder Complicating Pregnancy Patients with Different Severities" was published in 2022. Journal: Comput Math Methods Med.

### 3.3. Comparison of Blood Flow Parameters PI, RI, and S/D in Three Groups of UtA, UA, and MCA

The blood flow parameters PI, RI, S/D, and Qdv/Quv of UtA and UA were higher in the severe group than those in the control group and the mild group; the differences were all of statistical significance (*P* < 0.05) in Figures 4(a), 4(b), and 4(d). PI, RI, and S/D of MCA were lower in the severe group than those in the control group and mild group, suggesting the difference significant statistically (*P* < 0.05), shown in Figure 4(c).

In clinical practise, fetal UA blood flow measurements are crucial indicators of placental function alterations. Ciobanu et al. [23] found that for patients with abnormal UA blood flow resistance during pregnancy, the mean gestational age of delivery was significantly shortened after treatment, and the incidences of FIUD and neonatal asphyxia were significantly increased, even if the patients' UA resistance recovered to normal. The major blood artery supplying the cerebral hemisphere is the fetal MCA. Kim J et al. [24] come up with that RI of MCA had bidirectional changes; that is, the resistance decreased with hypoxia compensation and increased with decompensation. Among the cases here, blood flow parameters of MCA became decreased in the severe group, indicating that the MCA could reflect the severity of HDCP.

Changes in blood flow of UA are the earliest identifiable Doppler signals of early placental insufficiency. During normal fetal growth and development, the Qdv/Quv plays a vital role in regulating [22, 25, 26]. When the fetus is hypoxic, the DV dilates, the proportion of blood flow from UV into DV increases, and the Qdv/Quv increases sharply. Pinter et al. [27] suggested that fetal venous blood flow change was superior to arterial blood flow change in predicting adverse pregnancy outcomes. For cases in both the mild and the severe groups, the Qdv/Quv was increased compared with that of the normal control pregnant women, which was consistent with the description of the above research. Measurement of DV hemodynamics contributes to the understanding of the pathological state of the fetal circulation, deepening the understanding of hemodynamics in many fetal diseases.

### 3.4. Comparison of PI, RI, and S/D of UtA, UA, and MCA in Different Pregnancy Periods

In early pregnancy, no significant difference was observed in PI, RI, and S/D of UtA among the three groups (*P* > 0.05). All of PI, RI, and S/D increased first and then decreased in the early, middle, and later pregnancy in the severe group, with the difference significant statistically (*P* < 0.05). In the middle and later stages, those were higher than those in the mild and the control groups, as the differences were of statistical significance (*P* < 0.05). PI, RI, and S/D were gradually decreasing in the three stages of pregnancy in the control group, showing the significant differences statistically (*P* < 0.05) as presented in Figure 5.

The article "Fetal and Neonatal Middle Cerebral Artery Hemodynamic Changes and Significance under Ultrasound Detection in Hypertensive Disorder Complicating Pregnancy Patients with Different Severities" was published in 2022. Journal: Comput Math Methods Med.

The PI, RI, and S/D of UA in the middle and later stages of pregnancy declined steadily in both the mild and severe groups, with statistically significant differences (*P* 0.05). In the later stage, the severe group's PI, RI, and S/D were higher than the control group's, statistically and substantially (*P* 0.05) in Figure 6.

PI, RI, and S/D of MCA were all decreased gradually in the three groups in the middle and later pregnancy; the differences were also proved significant statistically (*P* < 0.05). Higher than those in the control group, PI, RI, and S/D were much different in the severe group in the middle and later stages statistically and significantly (*P* < 0.05), which are presented in Figure 7.

Under normal circumstances, blood flow parameters of UtA should go down gradually with gestational time. In this work, blood flow parameters PI, RI, and S/D of UtA gradually decreased with the increase of gestational age in the normal control group. But those increased first and decreased then from the early stage to the middle stage in the severe group, higher than those of the control group notably except in the early pregnancy (*P* < 0.05). With the development of embryos during normal pregnancy, placental trophoblast cells infiltrate continuously, UtA vascular remodelling is strengthened, the lumen is continuously enlarged, and the elasticity of the vascular wall is reduced. Uterine blood flow changes to low resistance and high flow rate from the high resistance and low flow rate before pregnancy [28–30]. The placental trophoblasts of pregnant women with HDCP have insufficient ability to infiltrate the arteries, the strength and quantity of vascular remodelling are also insufficient, the muscle layer of the vascular wall still maintains a large elasticity, and the vascular resistance goes up. PI, RI, and S/D values increase under the Doppler ultrasound quantitative analysis. The measurement of UA hemodynamic parameters can reflect the circulatory status between the fetus and the placenta. The results of this work demonstrated that the PI, RI, and S/D of UA increased abnormally in the control group in the middle and later stages of pregnancy. This indicated that the blood flow resistance of UA in HDCP patients was greater with less blood flow volume, because of the circulatory disorders in the fetus caused by the increased placental resistance.

The article "Fetal and Neonatal Middle Cerebral Artery Hemodynamic Changes and Significance under Ultrasound Detection in Hypertensive Disorder Complicating Pregnancy Patients with Different Severities" was published in 2022. Journal: Comput Math Methods Med.

### 3.5. Comparison of Fetal Pregnancy Outcomes

Among the 40 cases in the control group, there were 3 cases got abnormal pregnancy outcomes (including 2 cases with premature birth and 1 case with FGR); the incidence was 7.5%. In the mild group, 13 cases had abnormal pregnancy outcomes (11 cases of premature birth, 8 cases of FGR, 4 cases of FIUD, and 6 cases of neonatal asphyxia), with the incidence of 32.5%. In the severe group, 19 cases suffered from abnormal pregnancy outcomes (premature birth in 17 cases, FGR in 18 cases, FIUD in 13 cases, and neonatal asphyxia in 16 cases), working out an incidence of 47.50%. The incidence of abnormal pregnancy outcomes was higher markedly in the severe group than that in the mild and the control groups, suggesting the significant differences statistically (*P* < 0.05). Detailed data are shown in Table 2.

### 3.6. Comparison of Perinatal Prognosis

There were big statistical differences in the weeks of delivery, birth weight, pH value of UA, Apgar score, and placental weight of neonates among three groups (*P* < 0.05). Between the mild group and the control group, no statistical difference was found (*P* > 0.05) as displayed in Table 3.

The placenta's size is critical for supporting appropriate fetal growth. The weight of the placenta in the normal pregnancy group was substantially higher than that in the HDCP group, according to Esposito et al. [31]. The severe group had significantly lower weeks of delivery, placental weight, and neonatal birth weight than the normal and mild groups, which was consistent with the previous study. The reason may be that the total number of villi in the placenta increases with the weight of the placenta.

### 3.7. Blood Flow Parameters of UtA, UA, and MCA in the Diagnosis of Adverse Pregnancy Outcomes

Table 4 displays the AUC, appropriate cut-off value, sensitivity, and specificity of pregnancy outcomes, as well as UtA, MCA, and UA blood flow parameters. For the ROC curve, the optimal cut-off value of PI was 1.17, and the AUC was 0.78; the sensitivity and specificity were 80.2% and 72.1% for predicting adverse pregnancy outcomes, respectively. Of RI, the optimal cut-off value and AUC were 0.67 and 0.72, respectively; the sensitivity and specificity were 53.8% and 86.7%, respectively. Of S/D, the optimal cut-off value, AUC, sensitivity, and specificity were 2.68, 0.71, 78.3%, and 54.6%, respectively. PI had the most diagnostic value, as shown in Figure 8(a).

The appropriate cut-off value and AUC of PI were 0.95 and 0.82, respectively, with the ROC curve drawn by PI, RI, and S/D of UA as well as pregnancy outcomes; the sensitivity and specificity of PI for predicting bad pregnancy outcomes were 73.2 percent and 77.2 percent, respectively. The optimal cut-off value, AUC, sensitivity, and specificity of RI were 0.64, 0.76, 63.2%, and 75.8%, respectively. Those of S/D were 2.83, 0.68, 72.4%, and 68.3%, respectively. PI had the most diagnostic value of UA, which are shown in Figure 8(b).

The article "Fetal and Neonatal Middle Cerebral Artery Hemodynamic Changes and Significance under Ultrasound Detection in Hypertensive Disorder Complicating Pregnancy Patients with Different Severities" was published in 2022. Journal: Comput Math Methods Med.

With the ROC curve of MCA, the four indexes of PI were 1.67, 0.81, 68.7%, and 83.2%, respectively. Of RI, those were 0.68, 0.73, 89.4%, and 58.7%, respectively. Of S/D, those were 3.63, 0.86, 87.5%, and 78.6%, respectively. S/D showed the most diagnostic value of MCA, as it could be found in Figure 8(c).

The AUC was 0.98 in the ROC curve created by combining blood flow characteristics and pregnancy outcomes, and the sensitivity and specificity for predicting bad outcomes were 94.7 percent and 96.4 percent, respectively. When compared to a single blood flow parameter, the diagnostic value was higher, as illustrated in Figure 8(d).

Prasad et al. [32] reported that the continuous increase of UtA-PI predicted abnormal changes in vascular resistance, and dynamic monitoring of S/D could understand the uterine-placental circulation status. Elevated UtA-RI was the best predictor of severe FGR in high-risk groups, which illustrated that the blood flow parameters were complementary to each other and could evaluate and predict adverse pregnancy outcomes objectively.

## 4. Sensitivity and Specificity of the Combination of All Parameters in Diagnosing Adverse Pregnancy Outcomes

The combination of all the parameters showed the highest diagnostic value for FIUD, with an AUC of 0.89; its sensitivity and specificity were 86.3% and 88.4%, respectively. In this case, the AUC for FGR was 0.63, with the highest diagnostic sensitivity of 94.6%; but its specificity was a little lower, which reached 39.2% merely. These results are represented in Figure 9 and Table 5 in details.

### 4.1. Correlation between Fetal Hemodynamic Parameters and Poor Perinatal Prognosis

Logistic binary regression analysis was performed with the Qdv/Quv as well as hemodynamic parameters of UtA, UA, and MCA as independent variables, and whether an adverse perinatal outcome occurred was taken as the dependent variable. It was illustrated that poor perinatal prognosis was correlated with fetal Qdv/Quv as well as blood flow parameters PI, RI, and S/D of UtA, UA, and MCA (*P* < 0.05), as suggested in Table 6.

In correlation analysis, the poor perinatal prognosis was demonstrated to be correlated with fetal hemodynamic parameters of UtA, UA, and MCA and Qdv/Quv. These indexes could be auxiliary indexes for the evaluation of patients' condition and the prediction of perinatal prognosis, consistent with what was found by Maged et al. [33].

The article "Fetal and Neonatal Middle Cerebral Artery Hemodynamic Changes and Significance under Ultrasound Detection in Hypertensive Disorder Complicating Pregnancy Patients with Different Severities" was published in 2022. Journal: Comput Math Methods Med.

## 5. Conclusions

As the blood flow parameters of UtA, MCA, and UA in 120 pregnant women with singleton pregnancy were monitored and analysed, this work was aimed at exploring these blood flow parameters in HDCP patients and their correlations with pregnancy outcomes. Colour Doppler ultrasound could be utilised to detect PI, RI, and S/D of UtA, MCA, and UA in pregnant women, providing a baseline for measuring the fetus' intrauterine state and predicting negative pregnancy outcomes. The parameters in the later stage had the higher diagnostic value of adverse pregnancy outcomes. The combination of all the parameters could improve the diagnostic accuracy and provide a basis for guiding treatment and determining the best timing of delivery. The disadvantages of this research lay in that frequent fetal movement would affect the measurement of various parameters. The angle of the sampling between the sound beam and blood flow should be strictly required, and there might be slight errors. Furthermore, the sample size was small, resulting in some discrepancies in the results. In the future, larger sample sizes will be required for more complete studies and more valuable research outcomes. In conclusion, this work could provide reference for early prevention, early detection, and early treatment of HDCP, so as to improve adverse pregnancy outcomes.

## Figures and Tables

**Figure 1:** The blood flow spectra of fetal UtA. (a) Doppler waveform of UtA blood flow of pregnant women measured by transabdominal ultrasound in the control group. (b) Doppler waveform of abnormal UtA blood flow in the mild group. (c) Doppler waveform of abnormal UtA blood flow in the severe group. The red arrow indicated the diastolic notch.

**Figure 2:** Blood flow spectra of fetal MCA. (a) Doppler waveform of MCA blood flow in pregnant women under transabdominal ultrasound in the normal group. (b) Doppler waveform of abnormal MCA blood flow in the mild group. (c) Doppler waveform of MCA blood flow abnormality in the severe group.

**Figure 3:** Blood flow spectra of fetal UA measured by transabdominal ultrasound. (a) Doppler waveform of UA blood flow in the normal group. (b) Doppler waveform of abnormal UA blood flow in the mild group. Diastolic blood flow signal of UA disappeared. (c) Doppler waveform of abnormal UA blood flow in the severe group. The UA diastolic blood flow signal was reversed.

**Figure 4:** Comparison of fetal blood flow parameters. (a) Comparison of fetal blood flow parameters of UtA. (b) Comparison of those of UA. (c) Comparison of those of MCA. (d) Comparison of the fetal Qdv/Quv. Note: ∗ and △ marked the statistical differences in comparison with the normal and mild groups, respectively (*P* < 0.05).

The article "Fetal and Neonatal Middle Cerebral Artery Hemodynamic Changes and Significance under Ultrasound Detection in Hypertensive Disorder Complicating Pregnancy Patients with Different Severities" was published in 2022. Journal: Comput Math Methods Med.

**Figure 5:** Comparison of blood flow parameters PI, RI, and S/D of UtA in different stages. (a) PI comparison. (b) RI comparison. (c) S/D comparison. Note: ∗ and # indicated the significant difference statistically compared with the early and middle stages, respectively, *P* < 0.05.

**Figure 6:** Comparison of blood flow parameters PI, RI, and S/D of UA in different periods. (a) PI comparison. (b) RI comparison. (c) S/D comparison. Note: ∗ indicated there was a significant difference statistically compared with the early stage, while # indicated the same compared with those in the middle stage, *P* < 0.05.

**Figure 7:** Comparison of PI, RI, and S/D of MCA in different stages. (a) Comparison of PI. (b) Comparison of RI. (c) Comparison of S/D. Note: ∗ and # pointed out the differences significant statistically in comparison with those in the early and middle stages, respectively, *P* < 0.05.

**Figure 8:** ROC curves of UtA, MCA, and UA blood flow parameters as well as pregnancy outcomes. (a) ROC curves of UtA drawn under blood flow parameters and pregnancy outcomes. (b) ROC curves of UA. (c) ROC curves of MCA. (d) Blood flow parameter combined with pregnancy outcomes.

**Figure 9:** ROC curves drawn under the combined diagnosis with all parameters of adverse pregnancy outcomes.

**Table 1:** Comparison of the mean age and mean gestational age ($\bar{x}\pm s$).

Groups	Cases (*n*)	Mean age (years old)	Mean gestational age (weeks)
Control group	30	28.89 ± 2.360	32.67 ± 0.782
Mild group	30	27.68 ± 2.644	32.36 ± 0.563
Severe group	30	28.79 ± 2.571	32.61 ± 0.451

**Table 2:** Comparison of pregnancy outcomes of fetuses (*n*, %).

	Control group (*n* = 40)	Mild group (*n* = 40)	Severe group (*n* = 40)	*F*	*P*
Premature birth	2 (5)	11 (27.5)	17 (42.5)	8.37	0.002
FIUD	0	8 (20.0)	18 (45.0)	10.29	0.000
FGR	1 (2.5)	4 (10.1)	13 (32.5)	9.36	0.001
Neonatal asphyxia	0	6 (15.2)	16 (40.2)	11.37	0.000

**Table 3:** Comparison of perinatal prognosis (*n*, %).

	Control group (*n* = 40)	Mild group (*n* = 40)	Severe group (*n* = 40)	*F*	*P*
Weeks of delivery (weeks)	36.7 ± 3.2	33.2 ± 2.6	32.1 ± 2.5^∗^^△^	8.352	0.000
Birth weight (g)	2926.1 ± 634.3	2743.8 ± 73.2	2171.1 ± 745.3^∗^^△^	11.293	0.001
pH of UA	7.3 ± 0.1	7.1 ± 0.2	6.8 ± 0.1^∗^^△^	9.362	0.001
Apgar score (points)	10.0 ± 0.0	10.0 ± 0.0	8.3 ± 2.7^∗^^△^	10.281	0.002
Placental weight (g)	578.91 ± 132.6	553.2 ± 121.7	468.9 ± 102.4^∗^^△^	11.381	0.000

Note: ^∗^^△^ indicated that a difference significant statistically was shown compared with the control group and mild group, respectively, *P* < 0.05.

The article "Fetal and Neonatal Middle Cerebral Artery Hemodynamic Changes and Significance under Ultrasound Detection in Hypertensive Disorder Complicating Pregnancy Patients with Different Severities" was published in 2022. Journal: Comput Math Methods Med.

**Table 4:** AUC, optimal cut-off value, sensitivity, and specificity with blood flow parameters and pregnancy outcomes of UtA, MCA, and UA.

Test variables	AUC	Optimal cut-off value	Sensitivity (%)	Specificity (%)
UtA-PI	0.78	1.17	80.2	72.1
UtA-RI	0.72	0.67	53.8	86.7
UtA-S/D	0.71	2.68	78.3	54.6
UA-PI	0.82	0.95	73.2	77.2
UA-RI	0.76	0.64	63.2	75.8
UA-S/D	0.68	2.83	72.4	68.3
MCA-PI	0.81	1.67	68.7	83.2
MCA-RI	0.73	0.68	89.4	58.7
MCA-S/D	0.86	3.63	87.5	78.6
Combination of all parameters	0.98	/	94.7	96.4

**Table 5:** AUC, sensitivity, and specificity of the combined diagnosis for adverse pregnancy outcomes with UtA, UA, and MCA parameters.

Test variables	AUC	Sensitivity (%)	Specificity (%)
FIUD	0.89	86.3	88.4
Premature birth	0.72	89.2	51.2
FGR	0.63	94.6	39.2
Neonatal asphyxia	0.73	87.4	54.4

**Table 6:** Correlation between fetal hemodynamic parameters and poor perinatal prognosis.

Independent variables	*β*	Wald value	df	OR	*P*
Qdv/Quv	4.372	3.281	1	2.837	0.021
UtA-PI	2.271	4.872	1	3.782	0.001
UtA-RI	2.361	5.383	1	2.873	0.000
UtA-S/D	2.783	6.787	1	1.987	0.001
UA-PI	3.827	7.832	1	3.822	0.001
UA-RI	3.892	6.785	1	2.861	0.011
UA-S/D	2.371	7.684	1	0.563	0.002
MCA-PI	-1.982	7.982	1	0.462	0.004
MCA-RI	-4.381	6.483	1	0.632	0.006
MCA-S/D	-2.986	7.842	1	0.271	0.000

## Data Availability

The data used to support the findings of the study are included within the article.

## References

[1] Sinkey A., Battarbee N., Bello A., Ives C. W., Oparil S., Tita A. T. N. (2020). Prevention, diagnosis, and management of hypertensive disorders of pregnancy: a comparison of international guidelines. *Current Hypertension Reports*.

[2] Hauspurg M., Countouris J., Catov M. (2019). Hypertensive disorders of pregnancy and future maternal health: how can the evidence guide postpartum management?. *Current Hypertension Reports*.

[3] Behrens I., Basit S., Melbye M. (2017). Risk of post-pregnancy hypertension in women with a history of hypertensive disorders of pregnancy: nationwide cohort study. *BMJ*.

[4] Ukah U., de Silva D. A., Payne B. (2018). Prediction of adverse maternal outcomes from pre-eclampsia and other hypertensive disorders of pregnancy: a systematic review. *Pregnancy Hypertens*.

[5] Jones E., Hernandez T., Edmonds J., Ferranti E. P. (2019). Continued disparities in postpartum follow-up and screening among women with gestational diabetes and hypertensive disorders of pregnancy: a systematic review. *The Journal of Perinatal & Neonatal Nursing*.

[6] Gebremedhin A., Regan K., Ball S. (2021). Interpregnancy interval and hypertensive disorders of pregnancy: a population-based cohort study. *Paediatric and Perinatal Epidemiology*.

The article "Fetal and Neonatal Middle Cerebral Artery Hemodynamic Changes and Significance under Ultrasound Detection in Hypertensive Disorder Complicating Pregnancy Patients with Different Severities" was published in 2022. Journal: Comput Math Methods Med.

[7] Semmler J., Abdel-Azim S., Anzoategui S., Zhang H., Nicolaides K. H., Charakida M. (2021). Influence of birth weight on fetal cardiac indices at 35-37 weeks' gestation. *Ultrasound in Obstetrics & Gynecology*.

[8] Ali S., Heuving S., Kawooya M. (2021). Prognostic accuracy of antenatal Doppler ultrasound for adverse perinatal outcomes in low-income and middle-income countries: a systematic review. *BMJ Open*.

[9] Ayaz R., Günay T., Yardımcı D., Turgut A., Ankaralı H. (2021). The effect of 75-g oral glucose tolerance test on maternal and foetal Doppler parameters in healthy pregnancies: a cross-sectional observational study. *Journal of Obstetrics and Gynaecology*.

[10] Gómez-Roig M., Mazarico E., Cuadras D. (2021). Placental chemical elements concentration in small fetuses and its relationship with Doppler markers of placental function. *Placenta*.

[11] Monaghan C., Binder J., Thilaganathan B., Morales-Roselló J., Khalil A. (2018). Perinatal loss at term: role of uteroplacental and fetal Doppler assessment. *Ultrasound in Obstetrics & Gynecology*.

[12] Paules C., Youssef L., Rovira C. (2019). Distinctive patterns of placental lesions in pre-eclampsia vs small-for-gestational age and their association with fetoplacental Doppler. *Ultrasound in Obstetrics & Gynecology*.

[13] Wei Z., Mu M., Li M., Li J., Cui Y. (2021). Color Doppler ultrasound detection of hemodynamic changes in pregnant women with GDM and analysis of their influence on pregnancy outcomes. *American Journal of Translational Research*.

[14] Lee H., Lee S., Ko J., Kim S. J., Shin J. E. (2020). Association between fetoplacental Doppler results, placental pathology, and angiogenic factors among pregnant women with anxiety. *Taiwanese Journal of Obstetrics & Gynecology*.

[15] Roberts L., Ling H., Poon L., Nicolaides K. H., Kametas N. A. (2018). Maternal hemodynamics, fetal biometry and Doppler indices in pregnancies followed up for suspected fetal growth restriction. *Ultrasound in Obstetrics & Gynecology*.

[16] Ciobanu A., Rouvali A., Syngelaki A., Akolekar R., Nicolaides K. H. (2019). Prediction of small for gestational age neonates: screening by maternal factors, fetal biometry, and biomarkers at 35-37 weeks' gestation. *American Journal of Obstetrics and Gynecology*.

[17] Nader L., Zielinsky P., Naujorks A. (2018). Behaviour of the foramen ovale flow in fetuses with intrauterine growth restriction. *Obstetrics and Gynecology International*.

[18] Ton T., Bennett M., Incerti D. (2020). Maternal and infant adverse outcomes associated with mild and severe preeclampsia during the first year after delivery in the United States. *American Journal of Perinatology*.

The article "Fetal and Neonatal Middle Cerebral Artery Hemodynamic Changes and Significance under Ultrasound Detection in Hypertensive Disorder Complicating Pregnancy Patients with Different Severities" was published in 2022. Journal: Comput Math Methods Med.

[19] Martino D., Ferrazzi E., Garbin M. (2019). Multivariable evaluation of maternal hemodynamic profile in pregnancy complicated by fetal growth restriction: prospective study. *Ultrasound in Obstetrics & Gynecology*.

[20] Zijl M., Koullali B., Mol J., Snijders R. J., Kazemier B. M., Pajkrt E. (2020). The predictive capacity of uterine artery Doppler for preterm birth-a cohort study. *Acta Obstetricia et Gynecologica Scandinavica*.

[21] Liu H., Liu J. (2021). Improved support vector machine algorithm based on the influence of gestational diabetes mellitus on the outcome of perinatal outcome by ultrasound imaging. *Pakistan Journal of Medical Sciences*.

[22] Rubin J., Li S., Fowlkes J. (2021). Comparison of variations between spectral Doppler and Gaussian surface integration methods for umbilical vein blood volume flow. *Journal of Ultrasound in Medicine*.

[23] Ciobanu A., Wright A., Syngelaki A., Wright D., Akolekar R., Nicolaides K. H. (2019). Fetal Medicine Foundation reference ranges for umbilical artery and middle cerebral artery pulsatility index and cerebroplacental ratio. *Ultrasound in Obstetrics & Gynecology*.

[24] Kim J., Ha S., Jin W. (2021). Color Doppler ultrasonography for predicting the patency of anastomosis after superficial temporal to middle cerebral artery bypass surgery. *Acta Neurochirurgica*.

[25] Wu M., Lin Y., Lei F., Yang Y., Yu L., Liu X. (2021). Diagnostic value of prenatal ultrasound for detecting abnormal fetal blood flow. *American Journal of Translational Research*.

[26] Yin Q., Zhang Y., Ma Q., Gao L., Li P., Chen X. (2021). The clinical value of blood flow parameters of the umbilical artery and middle cerebral artery for assessing fetal distress. *American Journal of Translational Research*.

[27] Pinter S., Kripfgans O., Treadwell C., Kneitel A. W., Fowlkes J. B., Rubin J. M. (2018). Evaluation of umbilical vein blood volume flow in preeclampsia by angle-independent 3D sonography. *Journal of Ultrasound in Medicine*.

[28] Avitan T., Sanders A., Brain U., Rurak D., Oberlander T. F., Lim K. (2018). Variations from morning to afternoon of middle cerebral and umbilical artery blood flow, and fetal heart rate variability, and fetal characteristics in the normally developing fetus. *Journal of Clinical Ultrasound*.

[29] Herman H. G., Barber E., Gasnier R. (2018). Placental pathology and neonatal outcome in small for gestational age pregnancies with and without abnormal umbilical artery Doppler flow. *European Journal of Obstetrics, Gynecology, and Reproductive Biology*.

[30] Abdallah A., Eldorf A., Sallam S. (2019). Nuchal cord: impact of umbilical artery Doppler indices on intrapartum and neonatal outcomes: a prospective cohort study. *The Journal of Maternal-Fetal & Neonatal Medicine*.

The article "Fetal and Neonatal Middle Cerebral Artery Hemodynamic Changes and Significance under Ultrasound Detection in Hypertensive Disorder Complicating Pregnancy Patients with Different Severities" was published in 2022. Journal: Comput Math Methods Med.

[31] Esposito L., Salzano A., Russo M. (2020). Corpus luteum color Doppler ultrasound and pregnancy outcome in buffalo during the transitional period. *Animals (Basel)*.

[32] Prasad S., Goyal R., Kumar Y. (2017). The relationship between uterine artery two-dimensional color Doppler measurement and pregnancy outcome: a prospective observational study. *Journal of Reproduction & Infertility*.

[33] Maged A., Abdelaal H., Salah E. (2018). Prevalence and diagnostic accuracy of Doppler ultrasound of placenta accreta in Egypt. *The Journal of Maternal-Fetal & Neonatal Medicine*.

